The article "Performance of Emotional Cognition Education in College Students' Psychological Health Classroom" was retracted in 2023. Reasons: signs of a paper mill; suspected computer-generated content; unreliable results or conclusions; lack of ethics approval or compliance.

# Performance of Emotional Cognition Education in College Students' Psychological Health Classroom

**DOI:** 10.1155/2022/2802089

**Published:** 2022-08-31

**Authors:** Yinying Zheng, Xiaomin Yao, Yi Wang

**Affiliations:** ^1^College of Education,ZheJiang University, HangZhou 31000, China; ^2^Zhejiang University of Technology (ZJUT), HangZhou 310000, China; ^3^China Jiliang University, HangZhou 310018, China

## Abstract

With the development of modern technology, a variety of values and social thoughts based on streaming media have caused a huge impact on the field of ideology and culture, and contemporary college students are deeply affected. Nowadays, college students are very prone to problems such as lack of empathy, distorted values, and weakening of life values. College students commit suicide, homicide, and other illegal and criminal incidents due to unhealthy psychological reasons. This paper abstracts the emotional cognitive ability of college students into a psychological resilience model and then analyzes it. It is concluded that the overall applicability of college students to emotional cognition education in the psychological classroom is not high. In order to change the overall low applicability of this situation, this paper pioneers the application of the Internet of Things (IoT) technology to the emotional cognitive education system of college students' psychological classrooms. Through the experiment, four results of the two psychological classroom models were obtained under different genders, different grades, different household registration types, and comprehensive conditions. The improved mode of combining the Internet of Things technology with emotional cognitive education can increase the applicability of college students to emotional cognitive education in the psychological classroom by about 6.97%. It helps to cultivate and educate the positive emotions of college students and promote the comprehensive and healthy development of college students.

## 1. Introduction

Nowadays, scholars' research on emotional cognitive education in college students' psychological classrooms has certain limitations. Some researchers mainly used purely abstract theories such as educational psychology and hypothetical variable methods for research, with a lack of practice. Most of the methods used to study emotional cognition education are outdated and cannot play a good role in the rapidly changing modern teaching and modern society. Therefore, there is still a need for further systematic research on the problems and solutions of emotional cognitive education in college students' psychological classrooms.

Now, there are some studies on emotional cognitive education by scholars. Alar‒Zhan and other scholars explored the differential effects of different types and states of emotion and cognition in different regions of the brain. These differences are mainly reflected in the ability to respond, judgment, and decision-making. These findings have inspired educational researchers and provided a basis for their use in educational research [1]. The study by Yidana and others examined preservice teachers' levels of teaching engagement efficacy, as well as their behavioral, affective, and cognitive engagement efficacy. In addition, the sensitivity of their teaching participation efficiency to their demographic characteristics was also considered [2]. Research have been conducted highlighting the close relationship between executive functioning and the learning environment on campus. That is, an executive function creates the learning environment, and the learning environment in turn drives the development of an executive function. They believed that learning is a high cognitive function involving related aspects such as emotion, reward, self-efficacy, self-esteem, empathy, and value acquisition [3]. Falkstedt conducted experiments related to emotional cognitive education on hundreds of Swedes to explore the changes in cognitive and affective outcomes after long-term emotional cognitive education. Experiments showed that people, who have undergone long-term emotional cognitive education, have significant positive changes in this area [4]. Research by Read H and other scholars used affective cognitive education as part of comprehensive democratic education under current nonideal conditions to achieve broader social justice goals of promoting diversity, equity, and inclusion in public life [5]. Oliver and other scholars studied a quantitative comparison of action analog circuits in cognitive and affective empathy [6]. Yacoub and other scholars investigated a cognitive schema and emotion processing-based treatment regimen for reducing social anxiety among students in the field of elementary education [7].

The article "Performance of Emotional Cognition Education in College Students' Psychological Health Classroom" was retracted in 2023. Reasons: signs of a paper mill; suspected computer-generated content; unreliable results or conclusions; lack of ethics approval or compliance.

In addition, many scholars have studied the related factors of psychological classroom. Through experimental research, Wei and other scholars showed that college students, who completed the course of cross-cultural international psychology, can significantly improve their cross-cultural perception ability [8]. Research by Winston‒Proctor described a culturally responsive curriculum design model for teaching and learning at the core of undergraduate psychology courses. The results showed that after using the model, the teaching and learning efficiency of core content have been greatly improved [9]. In the study of Malik S E and other scholars, a perception model obtained by students in the psychological classroom was designed. The model can be used to explore the factors of students' perception in the psychological classroom [10]. The research of Peng and other scholars has shown that improving the level of computer science education and enhancing the ability of communication technology can contribute to the sustainable development of modern psychological classrooms [11]. Preliminary research by Roehling and other scholars showed that the good development of psychological classrooms has a positive impact on students' learning of science, technology, engineering, mathematics, and other courses, but has little impact on the heavy content of social science courses. The specific reason is that social science courses are biased toward liberal arts, and liberal arts students receive more abundant education in psychology courses [12]. Bernstein described a set of research strategies that can be widely used to assess the differences between new and traditional psychology courses [13]. Vitaro and other scholars discussed research on the neuropsychological classroom, in which some elements of the neuropsychological classroom can be deduced from the explanation of the psychological description process, assuming that the brain mechanism is ultimately sufficient to explain all psychological description phenomena. Then some elements of the neuropsychological classroom can be deduced through the explanation of the psychological description process [14]. Research by Nadelson and other scholars showed that teaching psychology in the classroom can be a challenging process, especially in the context of many conceptually complex, controversial, or counterintuitive content. Research showed that psychological classroom educators and psychological classroom education researchers need models to effectively solve difficult problems in teaching [15].

At the theoretical level, although some scholars have achieved good results in the field of emotional cognitive education and psychological classroom research and provided a certain and valuable reference for future research on emotional cognition education, research is still not comprehensive and complete. It is mainly reflected in the fact that the research methods are outdated, and there is a certain derailment from the current era. This paper mainly analyzes the performance of emotional cognition education in the psychological classroom of college students, drawing the conclusion that the applicability of emotional cognition education in the psychological classroom is not high for college students, and proposes countermeasures for this.

The article "Performance of Emotional Cognition Education in College Students' Psychological Health Classroom" was retracted in 2023. Reasons: signs of a paper mill; suspected computer-generated content; unreliable results or conclusions; lack of ethics approval or compliance.

## 2. Deconstruction and Coping Strategies of Emotional Cognitive Education Performance in College Students' Psychological Classroom

### 2.1. Necessity of Developing Emotional Cognition Education for College Students

The comprehensive development of college students' emotional cognition education is conducive to cultivating the positive and healthy psychology of college students. Good psychology is beneficial to the physical and mental health of college students, which is an important condition to ensure the normal development of functions and is the premise of improving learning efficiency. Therefore, improving the comprehensive quality of college students must be based on good psychological quality.

The all-around development of college students' emotional cognition education is conducive to exerting the potential of college students and promoting students' self-realization. Some studies suggest that the potential development of college students is determined by a variety of specific personality traits [16]. These personality traits include independence, sincerity, enthusiasm, etc. Emotional cognition education can enable college students with certain personality traits to have more complete personality traits, and enable college students, who do not have the above-mentioned personality traits to acquire these personality traits so that college students can better realize the unity of social value and self-value.

Studies have shown that most contemporary college students are the only seed in the family, favored by their elders, and have been in the core position of the family for a long time, so it is easy to breed many character weaknesses. In addition, college students are in restless adolescence, they have not yet gained social experience, and their values have not been perfected. When college students are confused or deviated in various aspects such as studies, love, social interaction, and employment, it will inevitably cause psychological fluctuations and negative emotions of college students. If this negative emotion is not resolved in a timely and effective manner, it will cause extreme reactions such as fear and pessimism, and then develop into mental diseases such as neurasthenia and anxiety, even leading to illegal and criminal incidents.

### 2.2. Deconstruction Framework of College Students' Emotional Cognitive Education Performance in Psychological Classroom

In the process of emotion regulation, cognition is a very important psychological process, and it is a cognitive way of managing events or information that can induce emotions. During this process, it is involved in the management of emotionally evoking events. In addition, information can be actively accessed through emotion-regulating cognition [17]. Cognition helps manage, regulate, and control emotions in response to stimuli. Affective cognitive regulation refers to changing a person's attention or evaluation of stimuli in a given situation to alter the intensity and duration of evoked emotions. Unlike the broad concept of emotion regulation, affective cognitive regulation is limited to self-regulation, an individual's conscious, cognitive reappraisal capacity [18].

The article "Performance of Emotional Cognition Education in College Students' Psychological Health Classroom" was retracted in 2023. Reasons: signs of a paper mill; suspected computer-generated content; unreliable results or conclusions; lack of ethics approval or compliance.

The adjustment of college students' affective cognition is affected by their range of activities and mode of activities. College students have a limited range of activities generally in the campus and its surrounding areas. The mode of activities is relatively monotonous, which leads to the fact that the adjustment of affective cognition is not spontaneous. It is necessary to carry out emotional cognitive education in the psychological classroom so that college students can use more positive and adaptive cognitive and emotional regulation, so as to improve their psychological resilience in the face of stress and maintain their mental health.

In this paper, the psychological resilience framework model is mainly used to analyze the emotional cognitive education performance of college students in the psychological classroom, as shown in Figure 1:

According to Figure 1, the analysis framework consists of four parts. Among them, students and teachers are general entities. Each constitutes a part, and teachers unilaterally output influence to students. The other part is to abstract the emotional cognitive education performance in college students' psychological classrooms into a psychological resilience model, so as to analyze it. The last part is to draw a conclusion after analysis, to classify the acceptance level of emotional cognition education in college students' psychological classrooms.

### 2.3. Attributes of Mental Resilience Model

#### 2.3.1. Concept of Resilience

Resilience has two core concepts: adversity and positive adaptation. To show resilience, it is necessary to place the object under investigation in an adversity environment and an adaptive environment, which is a key condition for evaluating a person's level of resilience. There are two key concepts of resilience: the pain period and the adaptation period [19]. Adversity and positive adjustment are important processes in demonstrating psychological resilience, which are key conditions for assessing a person's affective cognitive abilities. For most people, adversity is less about facing major hardships and more about the milder blows of everyday life. Another conceptual description of resilience revolves around the trait, consequential, and process theory of resilience [20]. Trait theory emphasizes that resilience is a relatively stable personality trait. Consequentialism emphasizes that individual resilience is a positive outcome of stress and adversity. Process theory regards resilience as a process in which individuals interact with their environment. The frame is shown in Figure 2:

Figure 2 shows the specific concept and process of psychological resilience. The entire framework is based on process theory, which provides a more comprehensive definition of resilience and helps researchers understand how resilience works, and suggest effective interventions. Consequentialism only focuses on the final positive results but ignores the process by that individuals achieve these positive results, which is not conducive to exploring the influencing factors and interventions of psychological resilience. Therefore, it is not adopted.

The article "Performance of Emotional Cognition Education in College Students' Psychological Health Classroom" was retracted in 2023. Reasons: signs of a paper mill; suspected computer-generated content; unreliable results or conclusions; lack of ethics approval or compliance.

In summary, this paper defines resilience as “an individual's ability to actively adapt to stressful situations in a threatening or challenging environment.” This stress refers not only to major life traumas but also to setbacks and challenges faced in daily life. Resilience is not a simple trait or outcome but the ability of an individual to continuously interact with the environment as a mental process. Therefore, in the process of abstracting college students' psychological resilience into a psychological resilience model, mainly examines the psychological self-healing ability of college students when they face major traumas and minor daily traumas in their lives.

#### 2.3.2. Influencing Factors of Psychological Resilience

Resilience is an important component of mental health, but there are also wide individual differences. Some individuals recover quickly after major trauma, and their level of mental health is even higher than before the trauma. Some people's mental health plummets after the trauma and never returns to baseline levels. Psychological resilience is influenced by the following factors:

Individuals with poor mental resilience are inherently affected. Animal experiments showed that mice born to mice that survived a nutrient-rich environment displayed less anxiety and were more flexible in coping with stress than mice born to a low-nutrient environment.

Risk factors are another factor that affects resilience. Risk factors often include potential negative outcomes, including both day-to-day ones and major ones. Risk factors are ubiquitous, and the negative effects of risk factors on individual development and function do not increase with the increase in number but increase in geometric progression. Therefore, the accumulation of adverse events can have a more severe impact on an individual's mental health and resilience.

The article "Performance of Emotional Cognition Education in College Students' Psychological Health Classroom" was retracted in 2023. Reasons: signs of a paper mill; suspected computer-generated content; unreliable results or conclusions; lack of ethics approval or compliance.

Another influencing factor related to resilience is protective factors, which can make individuals avoid or reduce the adverse effects of risk factors. Psychological resilience is the process of using protective factors to cope with adversity and actively adapt.

### 2.4. Psychological Resilience Model of Abstract Emotional Cognitive Ability of College Students

#### 2.4.1. Research Purpose

To analyze the current situation and characteristics of college students' psychological resilience, coping style, and mental health; to explore the relationship between mental resilience, coping style, and mental health of college students; to build a trajectory model of the impact of coping styles and resilience on mental health.

#### 2.4.2. Research Hypothesis

There are significant differences in resilience, coping styles, and mental health among different demographic variables. Resilience, mental health, and coping styles are intertwined. Resilience and mental health are reliable predictors of coping styles.

### 2.5. Coping Strategies Based on IoT Technology

By applying the Internet of Things technology to the emotional cognition education of college students' psychological classrooms, students can get richer educational resources, broader space, and more diverse channels. Therefore, in the process of carrying out the emotional cognition education of college students' psychological classroom, it is necessary to make full use of the network media, and actively explore new models and methods of college students' mental health education in combination with the actual situation and needs of college students in the current network environment. The coping strategy is shown in Figure 3:

It can be seen from Figure 3 that the coping strategy based on the Internet of Things technology consists of high-speed connection modules, security assurance modules, wireless network modules, and high-quality electronic teaching content. The formulation and implementation of this strategy follow the following principles:

#### 2.5.1. Principle of Comprehensiveness

This research constructs an indicator system based on the framework of the structure and process system of integrated learning, which is required to comprehensively cover all aspects of blended learning in teaching practice. Therefore, the indicator system should evaluate the key components of the integrated learning structure framework and process system as comprehensively as possible.

#### 2.5.2. Principle of Representativeness

When selecting specific indicators, targeted choices need to be made to ensure that the selected indicators are simple, complete, and accurate, and strive to select key indicators with strong representation. This prevents situations where too many metrics can affect observations.

The article "Performance of Emotional Cognition Education in College Students' Psychological Health Classroom" was retracted in 2023. Reasons: signs of a paper mill; suspected computer-generated content; unreliable results or conclusions; lack of ethics approval or compliance.

#### 2.5.3. Principle of Operability

The operating principle of the observation indicator is realized in the teaching practice of blended learning, and it is easy to observe. Metrics observed in blended learning, no matter whether they are qualitative or quantitative, must be quantifiable. Quantitative indicators (such as the number of teacher-student interactions) can be directly measured, and their data acquisition is relatively simple and easy. Quality metrics, such as the classroom environment, must be converted into performance metrics before they can be measured.

#### 2.5.4. Principles That Embody the Teaching and Learning Philosophy

The specific indicators in this paper are closely related to the concept of teaching and learning in the Internet of Things era, but focus on the observation indicators of traditional teaching. Focusing on the important items in the indicators, the concept of teaching and learning is explored through the properties of research indicators.

## 3. Coping Strategy Algorithm Based on Internet of Things Technology

Build a network based on IoT technology: it is assumed that there is a computationally intensive and latency-critical task that needs to be completed in a unit of time. The uploaded tasks are as formula (1):

(1) $$\begin{array}{c} T_{kn}=\left\{D_{kn},C_{kn},T_{kn}^{\text{max}}\right\}. \end{array}$$

In formula (1), *D*_*kn*_ indicates the amount of data uploaded by the task. *C*_*kn*_ represents the number of CPU cycles required by the server to process the task. *T*_*kn*_^max^ represents the maximum completion time allowed for the task.

Assuming a bandwidth of *B*_*S*_, the total transmission rate is as formula (2):

(2) $$\begin{array}{c} R^{S}=B_{s}{\text{log}}_{2}\left(1+\frac{G_{kn}^{S}P^{S}}{1+\sigma^{2}}\right). \end{array}$$

When intervening in the network, the transfer rate is as formula (3):

(3) $$\begin{array}{c} R_{kn}^{S}=a_{kn}R^{S}=a_{kn}{\text{log}}_{2}\left(1+\frac{G_{kn}^{S}P^{S}}{1+\sigma^{2}}\right). \end{array}$$

In formula (3), *G*_*kn*_^*S*^ means channel gain. *P*^*S*^ means transmit power. *σ*^2^ represents the noise power.

Corresponding transmission delay is as formula (4):

(4) $$\begin{array}{c} t_{kn}^{ST}=\frac{D_{kn}}{R_{kn}^{s}}=\frac{D_{kn}}{a_{kn}R^{S}}. \end{array}$$

The constraints are as formula (5):

(5) $$\begin{array}{c} e_{kn}^{S}=e_{kn}^{M}=e_{kn}^{C}=1. \end{array}$$

The server execution time is as formula (6):

(6) $$\begin{array}{c} t_{kn}^{E}=\frac{C_{kn}}{f_{kn}}. \end{array}$$

Among them, *f*_*kn*_ represents the CPU frequency allocated by the server.

The article "Performance of Emotional Cognition Education in College Students' Psychological Health Classroom" was retracted in 2023. Reasons: signs of a paper mill; suspected computer-generated content; unreliable results or conclusions; lack of ethics approval or compliance.

The task response time is as formula (7):

(7) $$\begin{array}{c} t_{kn}^{2}=t_{kn}^{ST}+t_{kn}^{ME}+T_{sm}. \end{array}$$

In formula (7), *T*_*sm*_ represents the transmission delay from base station to base station. *t*_*kn*_^*ME*^. represents the execution computation delay of the task in the data center.

When a task is assigned, it can be done so that all other tasks are finished as quickly as possible and that the most effective use of resources is made, in addition to guaranteeing that each task is finished before its assigned deadline. Because more resources are available to devote to the subsequent task when a task is completed as soon as possible and the subsequent batch of tasks arrives, as demonstrated by formula (8):

(8) $$\begin{array}{c} \text{min}\frac{1}{\sum_{n=1}^{N}k_{n}}\sum_{kn=1}^{N}\sum_{kn=1}^{kn}t_{kn}. \end{array}$$

There are four constraints as formulas (9)–(12):

(9) $$\begin{array}{c} t_{kn}\leq T_{kn}^{\text{MAX}},\;n\in N,\;kn\in K_{n}. \end{array}$$

(10) $$\begin{array}{c} \sum_{kn=1}^{kn}a_{kn}\leq 1. \end{array}$$

(11) $$\begin{array}{c} \sum_{kn=1}^{kn}e_{kn}^{S}f_{kn}\leq C_{S},\sum_{kn=1}^{N}\sum_{kn=1}^{kn}t_{kn}. \end{array}$$

(12) $$\begin{array}{c} b_{kn}\in \left\{0,1\right\},e_{kn}^{S}\in \left\{0,1\right\},e_{kn}^{M}\in \left\{0,1\right\},e_{kn}^{C}\in \left\{0,1\right\}. \end{array}$$

Among them, *t*_*kn*_ represents a constant related to the transmission distance, which is used to ensure that each task can be completed by the deadline. *a*_*kn*_ represents the sum of the percentage of wireless transmission slots.

The resource allocation problem is simplified to formula (13):

(13) $$\begin{array}{c} \underset{a,f}{\text{min}}T\left(\gamma^{0},a,f\right). \end{array}$$

The gradient operation is performed, and the derivation results are as formula (14):

(14) $$\begin{array}{c} \left(1-b_{kn}\right)\frac{-D_{kn}}{{\left(a_{kn}\right)}^{2}R^{S}}+b_{kn}\frac{-D_{kn}}{{\left(a_{kn}\right)}^{2}R^{M}}+\mu =0. \end{array}$$

After sorting, formula (15) can be obtained:

(15) $$\begin{array}{c} \frac{-D_{kn}}{{\left(a_{kn}\right)}^{2}}\left(\frac{1-b_{kn}}{R^{S}}+\frac{b_{kn}}{R^{M}}\right)+\mu =0, \end{array}$$

*b*_*kn*_/*R*^*M*^ is used to indicate that the computing resources allocated by each data center are less than or equal to the computing resources owned.

Case *μ*=0 can be excluded as formula (16):

(16) $$\begin{array}{c} \sum_{kn=1}^{kn}a_{kn}-1=0. \end{array}$$

Further formula (17) can be obtained:

(17) $$\begin{array}{c} a_{kn}=\sqrt{\frac{1}{\mu }D_{kn}\left(\frac{1-b_{kn}}{R^{S}}+\frac{b_{kn}}{R^{M}}\right)}. \end{array}$$

For the convenience of description, it can be simplified as formula (18):

(18) $$\begin{array}{c} a_{kn}=A_{kn}\sqrt{\frac{1}{\mu }}, \end{array}$$

*A*_*kn*_ is used to indicate that the task can only be offloaded to one data center for execution.

The article "Performance of Emotional Cognition Education in College Students' Psychological Health Classroom" was retracted in 2023. Reasons: signs of a paper mill; suspected computer-generated content; unreliable results or conclusions; lack of ethics approval or compliance.

Formula (18) is substituted to obtain formula (19):

(19) $$\begin{array}{c} \sum_{kn=1}^{K_{n}}A_{kn}\sqrt{\frac{1}{\mu }}-1=0. \end{array}$$

The radio resource allocation scheme can be obtained as formula (20):

(20) $$\begin{array}{c} a_{kn}=\frac{A_{kn}}{\sum_{kn=1}^{K_{n}}A_{kn}}. \end{array}$$

## 4. Experimental Deconstruction and Comparison of Emotional Cognitive Education Performance under Two Psychological Classroom Models

### 4.1. Research Samples

This paper selected undergraduate students from some schools and conducted an experimental investigation by randomly distributing questionnaires. A total of 500questionnaires were designed and prepared for the experimental investigation, and 468 valid questionnaires were available. The age range of the surveyed college students was 18 to 22 years old. The properties of the survey object are shown in Figure 4:

### 4.2. Research Process

The questionnaires have different types of questions for the two models of classrooms. One is in the traditional psychological classroom environment, and the other is in the Internet of Things psychological classroom environment. The test methods include field measurement and online filling. The steps to organize the questionnaire are as follows: First, the questionnaires with incomplete responses, questionnaires with no response content, questionnaires with unknown personal information, and questionnaires of extreme value types were screened out. Only valid questionnaires were retained; secondly, statistical quantitative mathematics software was used to carry out statistical analysis on valid data.

### 4.3. Experimental Test

All comparative analyses were based on questionnaire survey results to design scores to obtain an applicability score, which ranged from 1 to 5. The higher the score is, the stronger the applicability is.

#### 4.3.1. Differences in the Applicability of the Two Psychological Classroom Models for College Students under Different Genders

Under normal circumstances, college boys have relatively stable emotions and are more proactive and independent. They can adapt to the environment well. But at the same time, they are also aggressive. Compared with male college students, female college students are emotionally unstable, prone to sentimentality, lack of stamina or energy, and have poorer mental health. The differences in the applicability of the two psychological classroom models for college students of different genders are shown in Figure 5:

It can be seen from Figure 5 that the differences in the applicability of different genders under the same psychological classroom model are not obvious, but the applicability of college students' emotional cognition education under the improved psychological classroom model is significantly higher than that of the traditional psychological classroom model. This verifies that male college students have more stable emotional and psychological resilience than female college students.

The article "Performance of Emotional Cognition Education in College Students' Psychological Health Classroom" was retracted in 2023. Reasons: signs of a paper mill; suspected computer-generated content; unreliable results or conclusions; lack of ethics approval or compliance.

#### 4.3.2. Differences in the Applicability of the Two Psychological Classroom Models for College Students in Different Grades

The first-year students are in the adaptation stage. They have just graduated from high school and have a poor ability to regulate their emotions in the short term. Therefore, the emotional cognition education of students at this stage is particularly important. Sophomore students have basically adapted to the environment, which is a critical period for the gradual establishment of emotional cognition concepts. The third-year students' thinking is more mature, and their practicality, environmental adaptability, and psychological endurance have been enhanced. Senior students are facing graduation. They are under great pressure at this stage, but their psychological endurance has not been significantly weakened. The difference in applicability under different grades is shown in Figure 6:

It can be seen from Figure 6 that the applicability of different grades under the same psychological classroom model is quite different, and the applicability of freshmen is the worst. Under the traditional psychological classroom model, the questionnaire scores of the sophomore, junior, and senior students all reached four points or more, and only the freshman students scored less than four points. The applicability of a student is not high.

#### 4.3.3. Differences in the Applicability of the Two Psychological Classroom Models for College Students under Different Household Registration Types

Due to the differences in the living environment, growth experience, and education level of college students from rural families and urban families, students from rural families and students from urban families have different degrees and types of psychological problems and psychological pressures. Under normal circumstances, the psychological problems of rural students may be more likely to breed, and differences in economic conditions may be one of the reasons for psychological problems. The differences in applicability under different household registration types are shown in Figure 7:

As can be seen from Figure 7, the differences in the applicability of different household registration types under the same psychological classroom model are not obvious, and the improved psychological classroom model has little difference in the applicability of college students' emotional cognition education compared with the traditional psychological classroom model. There is a discrepancy between this result and general cognition, which may be greatly influenced by the subjectivity of individual choice.

The article "Performance of Emotional Cognition Education in College Students' Psychological Health Classroom" was retracted in 2023. Reasons: signs of a paper mill; suspected computer-generated content; unreliable results or conclusions; lack of ethics approval or compliance.

#### 4.3.4. Comprehensive Judgment of the Differences in the Applicability of College Students between the Two Psychological Classroom Models

The difference in applicability under comprehensive judgment is shown in Figure 8:

It can be seen from Figure 8 that under comprehensive consideration, the applicability of college students' emotional cognition education under the improved psychological classroom model is significantly higher than that of the traditional psychological classroom model, with an increase of about 6.97%. The results show that the improved emotional cognition education in the psychological classroom of college students is more suitable for students, which can have a better positive significance for the mental health of college students.

## 5. Conclusions

This paper uses the psychological resilience model to analyze the performance of emotional cognitive education in college students' psychological classrooms from four aspects and draws the conclusion that the overall applicability of college students' emotional cognitive education in psychological classrooms is not high. The application of the Internet of Things technology to the improvement of emotional cognitive education in college students' psychological classrooms can increase the applicability of college students' emotional cognitive education in psychological classrooms by about 6.97%. It provides the improvement direction and reference for the emotional cognition education of college students' psychological classrooms.

## Figures and Tables

**Figure 1:** An analysis framework for the educational performance of college students' emotional cognitive education.

**Figure 2:** Psychological resilience framework.

**Figure 3:** Coping strategies based on IoT technology.

**Figure 4:** Investigate student attributes.

**Figure 5:** Differences in the applicability of the two models in different genders.

**Figure 6:** Differences in the applicability of the two models in different grades.

**Figure 7:** Differences in the applicability of the two models under different household registration types.

**Figure 8:** Differences in applicability under comprehensive judgment.

The article "Performance of Emotional Cognition Education in College Students' Psychological Health Classroom" was retracted in 2023. Reasons: signs of a paper mill; suspected computer-generated content; unreliable results or conclusions; lack of ethics approval or compliance.

## Data Availability

The data used to support the findings of this study are available from the corresponding author upon request.
